The article "Growth of L-asparagine monohydrate organic single crystals: An experimental and DFT computational approach for nonlinear optical applications" was retracted in 2025. Reason: concerns about the citations.

# Growth of L-asparagine monohydrate organic single crystals: An experimental and DFT computational approach for nonlinear optical applications

**DOI:** 10.1016/j.heliyon.2024.e39842

**Published:** 2024-10-26

**Authors:** Md Anisur Rahman, Jiban Podder

**Affiliations:** a Department of Physics, Bangladesh University of Engineering and Technology, Dhaka, 1000, Bangladesh; b Department of Basic Sciences and Humanities (Physics), University of Asia Pacific, Dhaka, 1205, Bangladesh

**Keywords:** L-asparagine monohydrate, Structural investigation, Linear and nonlinear optical characteristics, HOMO-LUMO, Density functional theory

## Abstract

Good optical quality of L-asparagine monohydrate (C_4_H_8_N_2_O_3_.H_2_O) organic single crystal has been grown by adopting natural slow evaporation process at room temperature from aqueous solutions. The lattice parameters obtained by powder X-ray diffraction data revealed orthorhombic crystal system of the harvested crystal. The morphology and planes of the crystal have been identified. The molecular vibrations and functional groups have been specified by Fourier transform infrared (FTIR) spectroscopy studies. Energy dispersive X-ray (EDX) study has been availed to find out the elements constituting the crystal. Scanning electron microscopy, (SEM), provided the surface morphology of the crystal. The dependence of dielectric properties on frequency and temperature have been investigated and the electronic polarizability (α) has been determined. UV–vis spectral analysis shows that the crystal possesses good optical transmittance in the visible part of the energy spectrum. The optical band gap and the Urbach energy have been determined from lower absorption edge. Third order nonlinear susceptibility χ^(3)^, nonlinear refractive index (n_2_), and linear susceptibility χ^(1)^ have been calculated by Miller's generalized rule. The first-principle computation of band structure of electrons and the electron density of states have been discussed, which suggest that the crystals possess direct band gap. Density Functional Theory (DFT) with B3LYP function by Gaussian09W software was utilized to calculate HOMO-LUMO energy gap as well as non-linear optical parameters namely, linear polarizability (α), hyperpolarizability (β and γ) and dipole moment (μ) of L-asparagine monohydrate crystal. All the findings prove that L-asparagine monohydrate is a promising NLO crystal.

## Highlights

• Good quality L-asparagine monohydrate (C_4_H_8_N_2_O_3_.H_2_O) crystals have been grown by natural evaporation process.
• Third order nonlinear susceptibility χ^(3)^, linear susceptibility χ^(1)^ and nonlinear refractive index n_2_ have been calculated.
• The first-principles study of the electronic band structure and the electron density states have been discussed.
• Optical transparency and nonlinear optical susceptibility of L-asparagine monohydrate crystal indicates for opto-electronic and photonic applications.

## 1 Introduction

For the last several decades, nonlinear optical crystals have become the centre of interest for their unparallel optical properties for instance optical data storage, optical telecommunication, optical information processing and optical computing [1]. Organic materials possess substantial nonlinear susceptibilities in contrast to inorganic crystals, where α-amino acids have some unique features like weak hydrogen and van der Waals bonds, wide range of transparency in the visible and UV spectral regions, molecular chirality and zwitterionic property of the molecule [2,3]. The origin of nonlinear property in a crystal is the induced polarization at the time of interaction with high intensity electromagnetic field. Amino acids contain amino group (–NH_2_) and carboxyl group (–COOH), which act as protonated amino group (NH_3_^+^) (proton acceptor) and deprotonated carboxylic group (COO^−^) (proton donor) in solid state, that generates the required dipole behaviour for nonlinear activity to take place in a crystal [[4], [5], [6], [7], [8]]. L-Asparagine is one of the noteworthy organic amino acids showing orthorhombic crystal structure with non-centrosymmetric space group *P*2_1_2_1_2_1_. The unit cell parameters have the following values; a = 5.593 Å, b = 9.827 Å, c = 11.808 Å, and Z = 4 [9]. L-asparagine monohydrate (LAM) forms a complicated array of hydrogen bonds within asparagine molecules as well as between water and asparagine molecules [9,10]. These hydrogen bonds play a crucial role on the overall properties of organic crystals by creating additional attractive forces between molecules, and thus influencing the crystal structure, geometry, elasticity and optical properties. Recently, Sagane et al. [11] discussed effect of pH on properties of LAM crystal and reported improved linear and nonlinear optical properties of the crystal. Wlliam, D. et al. [12] investigated experimental as well as dipole moment, charge density, electrostatic potential, and electric field gradients in LAM crystal and opined for use of Hartree-Fock, and Density Functional Theory (DFT) method where experimental investigations are not possible, i.e., quantum chemical computations on amino acids make exact prediction of lots of electrostatic properties. F. Yogam et al. [9] also studied LAM crystal and reported low absorption in UV–vis region as well as SHG efficiency to be 7 times than that of KDP. Gupta et al. [13] determined optical transmittance, nonlinear absorption coefficient and nonlinear refractive index of the LAM crystal. Shakir et al. [14] found internal structural grain boundaries in their harvested LAM crystal, but the crystallinity improved significantly due to annealing at low temperature. Internal structural grain boundaries are the interfaces where two crystalline grains meet but orient in different directions and are formed due to temperature fluctuations during crystal growth. Suresh et al. [15] categorized their grown LAM crystal as soft material by microhardness study. Ramanadham et al. [16] discussed about the structure of LAM crystal by Neutron Diffraction. Thukral et al. [17] had grown LAM crystal and analyzed the optical property by photoluminescence, birefringence and Z-scan techniques.

As far as is known, no meticulous analysis on first principle calculation of density of states and band structure as well as HOMO-LUMO energy levels of LAM crystal highlighting NLO property have been made. Again, the morphology and planes of the harvested crystal have been obtained. In the present work, highly transparent LAM crystal has been harvested using natural slow evaporation technique and subjected to structural, morphological, optical, and dielectric studies. From the optical study, dielectric properties, band structure, HOMO-LUMO analysis and NLO properties have been discussed by DFT computation and inferred that the LAM crystal is a promising compound for nonlinear optical applications.

## 2 Crystal growth

For preparing solution, analar grade L-asparagine monohydrate (LAM) salt (of 99 % purity) was dissolved in double distilled water [[18], [19], [20], [21]]. The solution was stirred steadily for 10 h by magnetic stirrer (with hot plate facility), and was filtered using filter paper (Whatmann brand) before pouring into a beaker. The beaker was wrapped by porous sheet on the top to enable slow evaporation process to take place. Recrystallization technique was utilized to improve the quality of the crystals. Later, well-shaped and good quality seed crystals were selected, tied to a nylon thread and placed in a beaker containing saturated solution. After 30 days of natural evaporation, high quality transparent crystals were harvested as shown in Fig. 1 (i).

**Fig. 1:** (i) Image of as grown LAM crystal, (ii) Morphology with crystal planes of LAM crystal, (iii) Morphology of the grown crystal observed along the a axis.

## 3 Morphology of the crystal

Morphology with planes of LAM crystal obtained by WinXMorph software [22,23] is deepicted in Fig. 1 (ii) and (iii). The a axis is along 100 direction, b axis is along 010 direction and c axis passes through the intercept of 011 and 0 $\bar{\;1}\;1$ plane. A higher growth rate along the c axis is observed. Table 1 presents angle between different planes.

**Table 1:** Angle between different planes.

Plane	Angle	Plane	Angle	Plane	Angle	Plane	Angle	Plane	Angle
0 1 1	100.463°	0 $\bar{\;1}$$\bar{1}$	100.463°	0 $\bar{1}$ 1	39.768°	0 $\bar{1}$ 0	39.768°	0 1 1	39.768°
0 $\bar{\;1}\;1$		0 1 $\bar{1}$		0 $\bar{1}$ 0		0 $\bar{\;1}$$\bar{1}$		0 1 0	

## 4 Characterization process

### 4.1 General characterization

The crystallinity of the grown crystal has been studied by Philips X'Pert PW 3040 diffractometer with CuK_α1_ radiation (λ = 1.54 Å). A scintillation counter detected the diffracted X-rays, and the data were obtained in the 2-theta angle of 10–80° where the machine rotated with a step of 0.02°. Fourier Transform Infra-Red spectra were recorded by STA 449 F3 Jupiter spectrometer in the range of 4000 - 350 cm^−1^ by KBr pellet method. The surface of the LAM crystal was studied by scanning electron microscopy (JEOL JSM-7600F). The machine furnished with field emission (FE) facility (for obtaining high-resolution image) had been operated with accelerating voltage of 5 kV. The SEM was also equipped with energy-dispersive X-ray spectroscopy (EDS) facility in order to perform elemental analysis. Surface of the crystals were covered by thin carbon layer and imaging was conducted at highly vacuum state at room temperature. The crystals were dipped in water for 2 s to conduct etching study. The UV–Vis–IR spectrophotometer used in the present study was Shimadzu, UV-3100, Japan and the optical transmittance of the crystal (thickness = 2 mm) in the wavelength range of 190–1000 nm was studied. An impedance analyzer (Impedance Analyzer 41 92A LF) was utilized to assess the dielectric properties of the samples from 100 Hz to 1 MHz frequency range at various temperatures.

### 4.2 First-principles calculations

The plane-wave pseudopotential approach has been utilized in the first-principles calculation [24] which is based on density functional theory (DFT) with general gradient approximation (GGA) in the Perdew-Burke-Ernzerh (PBE) function [25]. In order to obtain optimized geometry of the unit cell, electronic band structure as well as electron density of states, the CASTEP program was availed [26]. The self-consistent field calculation has been utilized where the convergence criterion was 1 × 10^−6^ eV per atom. The plane-wave cut off energy was 400 eV. With the aim of attaining convergence of energy and sampling of the Brillouin zone of LA unit cell, the Monkhorst–Pack [27] k-point mesh 3 × 3 × 2 had been chosen for the electronic band structure calculation where the density was 0.07 Å^−1^ in the unit cell. The other parameters utilized in the calculation had been put to the default values of the CASTEP software module. The optimized unit cell is shown in Fig. 2 (ii).

**Fig. 2:** (i) Optimized molecular structure of LAM (for Gaussian 09W software), (ii) Optimized unit cell of LAM (for Materials Studio software).

### 4.3 Quantum chemical computation

The theoretical study was done by density functional theory (DFT) adopting Gaussian 09 software, where B3LYP function has been utilized and 6-31G∗ basis set has been employed. Gauss view suite was used to view the optimized geometry of the molecule. Fig. 2 (i) shows the optimized molecular structure.

## 5 Results and discussion

### 5.1 Structural characterization

Powder X-ray diffraction (PXRD) remains as a popular technique to investigate the crystallinity of a single crystal. From the obtained data and calculated lattice parameters, one can conclude that the grown single crystal possesses orthorhombic crystal structure with space group *P*2_1_2_1_2_1_. The XRD pattern of the powdered sample exhibited sharp and defined peaks revealing good crystallinity of the grown crystal (Fig. 3). The obtained results seem to be compatible with the reported values of literature. The refined cell parameters are well-matched with the standard CIF file (crystallographic information framework) collected from Crystallographic Open Data Base as given in Table 2. The small value of strain denotes little compressive strain in the crystal lattice. The phase refinement of the XRD data was conducted by Fullprof software (Fig. 4). The asymmetry function Pseudo-Voigt was adopted for modeling the peak profile function. Scale factor, cell parameters, overall B factor, background of the spectrum, shape parameters and atomic position were refined properly. The R-factor χ^2^ is the fitting factor of the experimental data. The R-factors representing the goodness of Rietveld refinement are the expected R‐factor R_exp_, the unweighted profile R-factor (R_p_), and the weighted profile R‐factor (R_wp_) which are tabulated in Table 2.

**Fig. 3:** XRD diffraction pattern of LAM along with reference pdf file.

**Table 2:** Calculated lattice constants, crystallite size, strain and fitting parameters of pure LAM crystal.

Sample	Lattice parameter (Å)			Volume (Å)^3^	Crystallite size D (nm)		Strain *ε* ( × 10^−3^)	R-factor
					W-H	Scherrer		
	a	b	c					
cif file reference code: (00-030-1529)	9.821	11.806	5.587	647.79				
LAM crystal	9.803	11.795	5.660	654.44	92.44	133.73	0.2	R_p_ = 9.67
								R_wp_ = 13.45
								R_exp_ = 10.35
								χ^2^ = 2.85

**Fig. 4:** Rietveld refinement of LAM crystal as carried out by FullProf software: the observed data are marked in red, calculated data in black, and difference plot in blue colour, and the inset is W-H plot of LAM xrd data. (For interpretation of the references to colour in this figure legend, the reader is referred to the Web version of this article.)

The crystallite size and strain existing in the crystal lattice can be evaluated using Williamson-Hall equation (W-H plot) [28]. The plot of β cosθ versus 4 sinθ is displayed in Fig. 4 (inset). The strain has been measured by drawing slope of the curve and the crystallite size has been calculated from the y-intercept (given in Table 2). As another option, the Scherrer equation (1) was adopted to find out the crystallite size [29,30].

(1) $$d=\frac{k\lambda }{\beta \;\cos\;\theta }$$

where, the full width at half maxima (FWHM) is *β*, Bragg diffraction angle is *θ*, Scherrer constant is *k*. A small difference is observed between the measured value of crystallite size by Scherrer equation and W-H plot. A slight change in peak intensity is observed possibly due to different crystallite size, instrumental factors (detector efficiency, X-ray beam intensity), absorption effects (due to composition), background scattering of the sample holder, temperature and atmospheric conditions [31].

### 5.2 FTIR analysis

Fig. 5 depicts the FT-IR spectra of LAM and the functional groups are given in Table 3. The peak observed at 3378 cm^−1^ denotes OH stretch of water and at 3102 cm^−1^ is the N–H vibration. The C–H bonding vibration is detected at 2924 cm^−1^. The small peaks prior to 2900 cm^−1^ are because of hydrogen bond between NH_3_^+^ and COO^−^ group. The asymmetric NH_3_^+^ deformation vibration occurs at 1632 cm^−1^. The peak seen at 1522 cm^−1^ might be owing to NH_2_ bending vibration. The CH_2_ deformation vibration give peaks at 1428 cm^−1^. The CH rocking vibration is seen at 1306 cm^−1^. The vibrations lying at 1234 cm^−1^ and 1148 cm^−1^ are due to NH_2_ in-plane rocking vibration and NH_3_^+^ rocking vibration respectively. The calculated bond lengths of various functional groups are provided in Table 4.

**Fig. 5:** Obtained FTIR spectra of LAM crystal.

**Table 3:** Vibrational frequency assignments.

Wave number (cm^−1^) in literature	Observed wave number (cm^−1^) for LAM	Assignments
3570–3200 [32]	3378	Stretching vibration of O-H
3500–3100 [33]	3102	N–H vibration in the molecule
2940–2840 [33]	2924	C – H bonding vibration in the molecule
Below 2900 [9]	Below 2924	Hydrogen bonding of NH_3_^+^ with COO^−^ grouping
1635–1585 [33]	1632	Asymmmetric NH_3_^+^ deformation vibration
1528 [34]	1522	NH_2_ bending vibration
∼1410 [33]	1428	CH_2_ deformation vibration
∼1325 [33]	1306	CH rocking vibration
∼1150 [33]	1234	NH_2_ in-plane rocking vibration
1149 [33]	1148	NH_3_^+^ rocking vibration
960–850 [32]	890	Hydrogen bonded O-H out-of-plane bending vibration
910–804 [33]	804	C-C stretching vibration
800-650 [33]	666	N-H Out-of-plane bending vibration
508 [35]	506	COO^−^ rocking vibration

**Table 4:** Reduced mass, force constant and bond length values of different functional groups of LAM.

Functional group	Reduced mass μ ( × 10^−27^ kg)	Observed FTIR peaks (cm^−1^)	Force constant k (N/cm)	Bond length r (Å) (From FTIR)	Bond length r (Å) (From Rietveld refinement)
OH	1.56	3378	6.3319	1.390	1.561
NH	1.55	3102	5.2950	1.475	1.657
CH	1.53	2924	4.6531	1.540	1.846
NH_2_	1.55	1522	1.2747	2.371	2.156
CH_2_	1.53	1428	1.1098	2.484	2.224
NH_3_^+^	1.55	1148	0.7252	2.862	2.348
CC	9.96	804	2.2867	1.952	1.482
COO^−^	11.4	506	1.0351	2.542	2.257

### 5.3 SEM and energy-dispersive X-ray spectroscopy (EDAX)

The study of SEM images gives visual information about surface morphology along with defects on the crystal surface. Fig. 6 (a) illustrates the SEM image of LAM. From the image, very fine parallel layer-like growth pattern is seen which reveals smoothness of the surface. The intrinsic structure of organic molecules forces them to stack in layers and intermolecular forces like hydrogen and van der Waals bond can generate layered growth during crystal growth [36]. Few micro crystals have been observed on the crystal surface which might be owing to temperature fluctuations or fast evaporation of water at the time of crystal growth. EDAX spectra as demonstrated in Fig. 6 (b) and Table 5, clearly reveals the constituent element of C, N and O of the grown LAM crystal in mass % and atom % and the stoichiometric ratio.

**Fig. 6:** (a) SEM image and (b) EDAX spectra of LAM crystal.

**Table 5:** Elemental composition of LAM.

Element	Mass %	Atom %	Stoichiometric%
C	15.17	23.95	20
N	03.38	04.57	10
O	81.45	71.48	20
H	–	–	50

Total =	100 %	100 %	100 %

### 5.4 UV–visible spectroscopy

UV–Vis spectral analysis is widely utilized to get the picture of optical transparency and other essential optical parameters of the grown crystal. If a material is to be used as NLO devices, the core demand is the lack of absorption in the wavelength range 350 nm–1100 nm. From Fig. 7 (a), it is seen that LAM crystal denotes 79.4 % transparency in the wavelength range 300–1000 nm and the lower cutoff occurs in ultraviolet region at wavelength 243 nm. This wavelength indicates shifting of an n orbital electron to anti-bonding π orbital [37].

**Fig. 7:** (a) UV–Vis spectra (b) (*αhν*)^2^ vs. photon energy for LAM crystals.

The negligible absorption and scattering behaviour of the amine group of LAM plays a key role in the transparency of the crystal (due to absence of strongly conjugated bonds) [38,39]. The absorption coefficient (α) can be measured from transmittance data as follows:

(2) $$\alpha =\frac{2.303}{d}\times \log\left(\frac{100}{\%T}\right)$$

where d symbolizes the thickness and log_10_ (1/T) denotes absorbance. In the region of high photon energy, the direct band gap value can be calculated from the Tauc's plot {Fig. 7 (b)} of energy dependence of absorption coefficient using the equation below:

(3) $$\alpha h\nu =A{\left(h\nu -E_{g}\right)}^{n}$$

where h symbolizes the Planck's constant, *ν* denotes the frequency of the incident photon, E_g_ represents optical bandgap energy and A is a constant. n denotes the type of electronic transition (n = 3/2 for forbidden direct transition, n = 3 for forbidden indirect transition, n = 2 for indirect transition and n = 1/2 for direct transition). Taking logarithm of equation (3) and differentiating with respect to hυ, we arrive at the equation as follows:

(4) $$\ln\left(\alpha h\nu \right)=\ln\left(A\right)+n\;\ln\left(h\nu -E_{g}\right)$$

(5) $$\frac{d\left[\ln\;\left(\alpha h\nu \right)\right]}{d\left(h\nu \right)}=\frac{m}{\left(h\nu -E_{g}\right)}$$

Fig. 8 (a) shows the graph plotted between [ln(αhυ)]/hυ and hυ from which the value of E_g_ can be estimated. The discontinuity in the curve provides information on single [40] as well as multiple [41] stage optical transitions.

**Fig. 8:** (a) Graph of [ln (αhυ)]/hυ vs. hυ, (b) graph of [ln (αhυ)] vs. [ln (hυ - Eg)].

In the current study, an optical transition having single stage with discontinuity exists at a specific value of knee point (E_g_ = 4.99 eV). The value of n is calculated from the graph of ln(αhυ) vs ln(hυ-E_g_) and it is measured as 0.457 ≈ 0.5 ≈ 1/2 (slope of the linear fit) as shown in Fig. 8 (b). It substantiates the direct band gap nature in optical transition of LAM crystal. From theoretical point of view, the optical band gap can also be measured by the following equation:

(6) $$E_{th}=\frac{hc}{\lambda_{\max}\left(nm\right)}$$

where *λ*_max_ represents cutoff wavelength (243 nm) and c symbolizes the velocity of light. From equation (6), the energy band gap has been calculated as 5.11 eV that is very close to the value obtained from experiment. So, it can be concluded that the large transmission at visible spectrum and the lower cutoff wavelength at ultraviolet range confirms for optoelectronic and photonic device applications [42,43].

#### 5.4.1 Determination of Urbach energy

In the curve of absorption coefficient, the observed exponential portion close to the edge of optical band termed as Urbach tail exits. This exponential tail extends more in solids having poor crystalline structure and amorphous solids. If this tail seems to be minimal, then it denotes good crystallinity of the material [[44], [45]]. The Urbach empirical rule is as follows [46]:

(7) $$\alpha =\alpha_{0}\;\exp\left(\frac{h\nu }{E_{U}}\right)$$

where α_0_ denotes a constant and E_U_ represents Urbach energy. Considering logarithm for whole of equation (7), we can obtain the following equation:

(8) $$\ln\;\alpha =\ln\;\alpha_{0}+\left(\frac{h\nu }{E_{U}}\right)$$

when a graph (Fig. 9 a) is plotted between ln (α) and incident photon energy (hυ), the Urbach energy (E_U_) is determined from the inverse of the slope of the linear fit. The value of E_U_ has been estimated to be 0.192 eV. This value indicates the range up to which the fluctuation of optical band gap of the crystal might extend i.e. up to ±0.192 eV (E_u_ = E_u1_ + E_u2_ in Fig. 9 b). This small value of E_U_ denotes that the LAM crystal possesses well crystalline structure and little disorder close to the band edge as well. Both the Urbach energy and the width of localized tail states (E_u1_ and E_u2_ in Fig. 9 b) at the energy bandgap edges are vital for gaining insight of the electronic nature of the material. Transition of electrons between the extended and localized states of the two bands in the forbidden band-gap is the cause for absorption spectra. Localized states are also termed as band tail states that arise owing to disorder of the material and spread between the band-gap region, lying beneath the conduction band or over the valence band (Fig. 9 b).

**Fig. 9:** (a) Plot of ln α vs photon energy for LA crystal, (b) Urbach band tail energy (E_U_) diagram.

In contrast, extended states are the electronic states that extend largely across the crystal lattice, forming the conduction and valence bands. The interaction between extended and localized band tail states shapes the absorption and electronic property of the material and thus gives precious understanding of the optical and electrical characteristics [[47], [48], [49]].

Urbach proposed one more equation for relating optical band gap energy and absorption coefficient as follows:

(9) $$\alpha =\beta \;\exp\left[\frac{\sigma \left(h\nu -E_{0}\right)}{K_{B}T}\right]$$

where β symbolizes a constant and σ is known as steepness parameter. For direct allowed transition, the transition energy E_0_ is considered equal to E_g_. However, for indirect transition, it equals E_g_ ± E_p_, where E_p_ stands for the energy of the phonon, arising owing to thermal dissociation in the lattice. As LAM crystal possess direct band gap energy, therefore, E_g_ = E_0_. If one takes logarithm of both sides of equation (12), it turns out as follows:

(10) $$\ln\;\alpha =\left(\ln\;\beta -\frac{\sigma E_{g}}{K_{B}T}\right)+\left(\frac{\sigma \left(h\nu \right)}{K_{B}T}\right)$$

Comparing equations (8), (10),

(11) $$\ln\left(\alpha_{0}\right)=\left(\ln\;\beta -\frac{\sigma E_{g}}{K_{B}T}\right)$$

and

(12) $$\left(\frac{h\nu }{E_{U}}\right)=\left(\frac{\sigma \left(h\nu \right)}{K_{B}T}\right)$$

where, E_U_ is 0.268 eV, T is equal to 273.16 K and K_B_ denotes the Boltzmann constant. The steepness parameter (σ) may be calculated from the equation below:

(13) $$\sigma =\left(\frac{K_{B}T}{E_{U}}\right)$$

The value of σ was determined to be 0.088. The electron-phonon interaction (E_e-p_) strength can be measured from the relation below [50]:

(14) $$E_{e-p}=\frac{2}{3\sigma }$$

The electron-phonon interaction (E_e-p_) strength has been estimated as 7.59 (Table 6).

**Table 6:** Optical constants of LAM crystal.

Optical Parameters	LAM	Reported value for LAM
Optical transparency	79.4 %	80 % [13]
Transparency cut-off	243 nm	240 nm [13]
E_g_ (eV)	5.00	5.09 [13]
E_th_ (eV)	5.11	˗
E_g_ (eV) (from band structure)	4.3	
E_g_ (eV) (from HOMO-LUMO)	5.03	
E_u_ (eV)	0.268	0.19 [11]
σ	0.088	˗
E_e-p_ (eV)	7.59	˗
χ^(1)^ (esu)	0.118	˗
n_2_ (m^2^/W)	7.85 × 10^−13^	5.44 × 10^−13^ [11]
χ^(3)^ (esu)	3.28 × 10^−14^	˗

#### 5.4.2 Dispersion of the refractive index

Reflectance (R) and Refractive index (n) have been determined using the relations below:

(15) $$R=\frac{1\pm \sqrt{1-\exp\;\left(-\alpha d+\exp\left(\alpha d\right)\right)}}{1+\exp\left(-\alpha d\right)}$$

and

(16) $$n=-\frac{\left(R+1\right)\pm \sqrt{3R^{2}+10R-3}}{2\left(R-1\right)}$$

Fig. 10 (a) shows dependence of refractive index on wavelength. The dispersion has been investigated by the single oscillator model proposed by Wemple and Di-Domenico (WDD) [51]. According to this model, the WDD equation is as follows

(17) $$n^{2}\left(h\nu \right)=1+\frac{E_{d}E_{0}}{E_{0}^{2}-{\left(h\nu \right)}^{2}}$$

Here, E_d_ and E_o_ are the strength (dispersion energy) and single oscillator energy respectively. The WDD equation can be simplified to:

(18) $${\left(n^{2}-1\right)}^{-1}=\frac{E_{0}}{E_{d}}-\frac{{\left(h\nu \right)}^{2}}{E_{0}E_{d}}$$

From the plot of (n^2^ − 1)^−1^ with (hν)^2^, the value of E_0_ and E_d_ have been calculated from the intercept over the vertical axis $\frac{E_{0}}{E_{d}}$ and slope (E_0_E_d_)^−1^ as shown in Fig. 10 (b).

**Fig. 10:** Plots of (a) Refractive index vs wavelength, (b) (n^2^ - 1)^−1^ vs (hν)^2^.

#### 5.4.3 Nonlinear optical properties

NLO crystals upon interacting with radiation might generate second and third harmonic effects. Second and third harmonic effects occur by the interaction of applied electric field (E) with the induced polarization (P). At low intensity, a linear optical effect is seen in the material as this interaction is a linear function; however at high intensity, nonlinear optical effects generate as the interaction is nonlinear function. Nonlinear optical parameters are related to the polarizability (P) as follows [52]:

(19) $$P=\chi^{\left(1\right)}E+\chi^{\left(2\right)}E^{2}+\chi^{\left(3\right)}E^{3}$$

where P symbolizes polarizability, χ^(1)^ represents linear optical susceptibility and χ^(2)^ and χ^(3)^ denote second and third order nonlinear optical susceptibilities, respectively. Generalized empirical relation Miller's rule is popularly utilized to predict third order nonlinear susceptibility (χ^(3)^) and nonlinear refractive index (n_2_). It is used extensively for finding new nonlinear optical crystals [53]. The optical linear susceptibility (χ^(1)^) may be calculated by eq. (23) [54]:

(20) $$\chi^{\left(1\right)}=\frac{n^{2}-1}{4\pi }$$

(21) $$\text{At}\;\text{infinite}\;\text{wavelength},\left(h\upsilon \to 0\right),n^{2}=1+\frac{E_{d}}{E_{0}}$$

Here, E_0_ and E_d_ denote single oscillator energy and dispersion energy respectively.

(22) $$\text{Hence}\;\chi^{\left(1\right)}=\frac{E_{d}}{4\pi E_{0}}$$

At long wavelength $(h\upsilon \to 0\;\text{and}\;n\to n_{0}$), χ^(3)^ and n_2_ can be measured from χ^(1)^ using Miller's rule [51]

(23) $$\chi^{\left(3\right)}=A\times {\left(\chi^{\left(1\right)}\right)}^{4}$$

(24) $$n_{2}=\frac{12\pi \chi^{\left(3\right)}}{n_{0}}$$

where the frequency independent constant A is equal to 1.7 × 10^−10^ esu. The values of χ^(1)^, χ^(3)^ and n_2_ are provided in Table 6.The higher order of crystallinity and the purity of the crystal can reduce losses due to scattering and defects that result in changing its nonlinear refractive index by modifying the local electric fields and polarizability. This leads to improve nonlinear optical response [55]. As the value of χ^(3)^ (3.28 × 10^−14^ esu) is almost same of the standard reference material KDP, the synthesized crystal can be a prospective candidate for optoelectronic and NLO devices.

### 5.5 Dielectric studies

The dielectric studies are critical for the investigation of defects and electrical characteristics in the material [56]. Molecular anisotropy, electronic polarization in the crystal and lattice dynamics can also be described explicitly from dielectric studies [57]. The dielectric permittivity was measured from the equation below:

(25) $$\text{Dielectric}\;\text{constant},\epsilon_{r}=\frac{C_{p}d}{\epsilon_{0}A}$$

The dielectric constant, ε_r_ and dielectric loss (tan δ) had been plotted with log f and at three temperature range (303 K, 323 K, 373 K) are illustrated in Fig. 11(a) and (b). Both the ε_r_ and tan δ maintain relatively larger values in the low frequency range and starts dropping with the rise of applied frequency but retain almost constant value in the high frequency, which is normal dielectric nature [58]. The high value of ε_r_ and tan δ at low frequency is contributed due to 4 polarizations, termed as, electronic, ionic, orientational and space charge polarizations [59]. The space charge being unable to keep up with the applied field with increasing frequency, results in decreasing values of ε_r_ and tan δ. The gradual decline in ε_r_ is an obvious sign that there exists fluctuating relaxation times and different sized domains in LAM crystal. The smaller value of dielectric constant of LAM crystal meets the critical condition for its application in SHG devices [60]. The small dielectric loss obtained for LAM crystal suggests that it has less defects and reveals its high optical quality and NLO applicability [61,62]. Nevertheless, these crystals are not appropriate for device applications below 1 kHz as the values are extremely large and at the same time unsteady due to all the four types of polarization [63]. In Fig. 11 (a), the dielectric constant is seen to rise with temperature that occurs owing to hopping mechanism of charge carriers by thermal excitation in the crystal lattice [64].

**Fig. 11:** Plot of (a) dielectric constant ε_r_ with log f and (b) dielectric loss (tan δ) with log f of LAM crystal.

#### 5.5.1 Deduction of solid-state parameters

According to theoretical calculation, the dielectric permittivity is dependent on all the atomic valence electrons of the molecule constituting crystal. The Penn gap and Clausius-Mosotti relation can be used to study the non-linear behavior a crystal using electronic polarizability α [65]. The valence electron plasma energy could be expressed as [66]:

(26) $$\hbar \omega_{p}=28.8\sqrt{\frac{Z\rho }{M}}$$

where Z denotes the total number of valence electrons (60) of the molecule, density is *ρ* = 1.569 gm/cm^3^ [17], *M* denotes the molecular mass (150 g/mol) and *ω*_*p*_ denotes plasma angular frequency. The dielectric constant measured at 1 MHz (*ε*_∞_) = 24.11. From Penn model [67], the average energy gap is calculated by the relation below:

(27) $$E_{p}=\frac{\hbar \omega_{p}}{\sqrt{\left(\varepsilon_{r}-1\right)}}$$

and the Fermi energy is

(28) Ef=0.2948(ℏωp)43

Finally, the electronic polarizability (α) has been estimated by the relation as follows [67,68]:

(29) $$\alpha =\left[\frac{{\left(\hbar \omega_{p}\right)}^{2}S_{0}}{{\left(\hbar \omega_{p}\right)}^{2}S_{0}+3E_{p}^{2}}\right]\frac{M}{\rho }\times 0.396\times 10^{-24}{cm}^{3}$$

where the constant S_0_ (dependent on particular material) was calculated by the equation below:

(30) $$S_{0}=1-\left[\frac{E_{p}}{4E_{f}}\right]+\frac{1}{3}{\left[\frac{E_{p}}{4E_{f}}\right]}^{2}$$

In another approach, the polarizability (α) has been evaluated by Clausius–Mossotti analysis as

(31) $$\alpha =\frac{3M}{4\pi N_{a}\rho }\left(\frac{\epsilon_{r}-1}{\varepsilon_{r}+2}\right)$$

where N_a_ denotes the Avogadro constant. The measured solid state parameters have been given in Table 7. As is observed that the value of the α of LAM crystal is 1.56 times greater than the standard NLO crystal KDP and proves the LAM crystal a prominent NLO material for application in photonics devices [69]. Considering the fact that the SHG efficiency depends on polarizability, it can be inferred that the SHG efficiency ought to be 1.56 times larger than that of KDP [69]. The plausible explanation for this greater value of α is the higher number of electron clouds as well as higher distance of electrons from the nuclear charge (when electrons are loosely connected to nuclear charge, it might result into enhanced polarizability in the crystal).

**Table 7:** Electronic polarizability parameters of LAM crystal.

Parameters	Present study LAM	Reported value (LAM) [17]
Electron plasma energy ђω_p_ (eV)	22.816	22.805
Penn gap energy E_p_ (eV)	4.746	6.0266
Fermi energy E_f_ (eV)	19.077	18.868
Polarizability α (Penn-gap Analysis) cm^3^ ( × 10^−23^)	3.33	3.4775
Polarizability α (Clausius–Mosotti equation) cm^3^ ( × 10^−23^)	3.36	3.329

### 5.6 Electronic band structures and density of states

The electronic states near the band gap dominates the optical characteristics in the visible and UV spectra of a crystal and very fundamental to analyze the cause of optical properties [70]. The dispersion of band structure in conjunction with the lines of high symmetry points of the Brillouin zone (BZ) is depicted in Fig. 12 (a). The Fermi level is seen at 0 eV on the energy scale as is evident from Fig. 12 (a).

**Fig. 12:** (a) The computed band structures and (b) the Brillouin zone of LA unit cell.

It is clear from the figure that the valence band (VB) maximum and the conduction band (CB) minimum is situated along C (k-points) indicating direct band gap nature of the crystal. The computed band gap value is 4.3 eV, which is lower than the experimentally obtained value 5.00 eV. This happens due to the reason that a discontinuity occurs in the derivative of the exchange–correlation energy while computation by density-functional theory. In DFT method, the calculated energy bandgap values are underestimated [71].

The partial densities of states (PDOS) along with the total density have been depicted in Fig. 13. The valence bands around −20 eV occurs due to 2s orbitals for oxygen (O), 2s orbitals for nitrogen (N), 1s orbital of hydrogen (H) and 2s orbitals for carbon (C). In the range −16 to −10 eV, strong hybridization is observed between N-2s and 2p orbitals as well as C-2s and 2p orbitals. The area ranging from −10 to −2 eV happens due to of 2p orbitals of O, 2p orbitals of N, and 2p orbitals of C. The contribution of the top of the valence band mainly comes from O-2p and N-2p orbitals. The unoccupied 2p orbitals of O, N and C atoms govern the bottom of the CB, where a little contribution from 1s orbital of H is also observed. Therefore, the absorption spectrum close to the UV–Visible cut-off wavelength may be regarded as the charge transfer from O-p and N-p states beneat the Fermi level to the mainly C-p states as well as mixing of O-p, N-p and H-s states.

**Fig. 13:** Analysis of the DOS and PDOS of s- and p-orbital contributions.

### 5.7 Frontier molecular orbital/HOMO-LUMO study

In quantum chemistry, the highest occupied molecular orbital (HOMO) and lowest unoccupied molecular orbital (LUMO) determine the bonding behaviour of the molecule. The LUMO and HOMO energies specify the electron-absorbing and releasing capacity of a molecule respectively. Both the HOMO and LUMO level are largely situated on the π-system of carboxyl and amino group of LAM, as is obvious from Fig. 14. The computed HOMO and LUMO energies are −8.39 eV and – 3.36 eV respectively for LAM molecule and the energy gap is 5.03 eV. Crystals having band gap values more than 3eV are suitable for UV and deep UV NLO applications. This band gap values prevent two-photon absorption making the crystal highly transparent in the UV region, and suitable for devices like UV lasers, frequency doubles, etc. [72].

**Fig. 14:** Frontier molecular orbital surfaces for the HOMO and LUMO plot of LAM molecule.

The global reactivity parameters have been attained from HOMO and LUMO energy by the following formulas using Koopmans theorem [[73], [74], [75], [76]] and given in Table 8:

(32) $$\text{Ionization}\;\text{energy},IE=-E_{HOMO}$$

(33) $$\text{Electron}\;\text{affinity},EA=-E_{LUMO}$$

(34) Hardness,η=(IE−EA)/2

(35) Chemicalpotential,μ=−(IE+EA)/2

(36) $$\text{Softness},S=\frac{1}{\left(2\eta \right)}$$

(37) Electronegativity,χ=(IE+EA)/2

(38) $$\text{Electrophilicity}\;\text{index},\omega =\mu^{2}S$$

**Table 8:** HOMO–LUMO parameters of LAM.

E_HOMO_ (eV)	E_HOMO_ (eV)	IE (eV)	EA (eV)	η (eV)	μ (eV)	S (eV)	χ (eV)	ω (eV)
−8.39	−3.36	8.39	3.36	2.515	−5.875	0.199	5.875	6.862

The HOMO energy is connected with the ionization energy (IE) and the LUMO energy is linked to the electron affinity during molecular interactions. The electrophilicity index measures energy stabilization, electronegativity index gives the tendency of a molecule to gain or lose electrons, chemical hardness measures the resistance to changes in electron distribution, i.e. the reactive tendency of the molecule.

#### 5.7.1 Molecular electrostatic surface potential (MEP) analysis

In molecules, the zone where partial charges are most likely to exist represents electronegativity of the atoms. The larger the difference in partial charges, the more polarizable the molecule is. The perfect visual tool MEP is used to illustrate the relative polarity of a molecule by showing the total density on electrostatic potential energy surface. On MEP surface, the blue area represents positive electrostatic potential known as nucleophilic site whereas and red denotes negative electrostatic potential known as electrophilic site. The green is the area of zero potential. When the colour is lighter or there is no colour at all on the surface, the molecule is non-polar in nature. The potential energy intensifies in the order of colour as follows: red < orange < yellow < green < blue. Fig. 14 depicts the MEP surface obtained by Gauss View software with iso-value of 0.0004 a.u. As is observed in Fig. 15, positive regions (blue) were identified on the hydrogen molecules whereas the negative area (red) is seen around the oxygen atom of LAM molecule. Some of the carbon atoms are situated in the green area denoting zero potential. Two apparent areas of nucleophilic and electrophilic attack sites are evident on the MEP surface map for LAM molecule.

**Fig. 15:** MEP map of a LAM molecule.

#### 5.7.2 Computational NLO studies

Quantum chemical computation is critical for understanding the connection between electronic structure of a molecule and its NLO response [77]. This computational method provides a cost-effective mean of designing molecular structure and predicting its NLO properties before synthesis. The polarizability α and first order hyperpolarizability β represent the range up to which the molecular electronic distribution of a is distorted by the applied electric field [78]. In the molecules, the strength of intermolecular charge transfer is known as β that creates NLO susceptibility in the material and is represented by the first order hyperpolarizability. The non-linear optical parameters had been computed using following equations [79] and given in Table 9:

(39) Dipolemoment,μ=(μx2+μy2+μz2)12

(40) $$\text{Polarizability},\alpha =\frac{\left(\alpha_{xx}+\alpha_{yy}+\alpha_{zz}\right)}{3}$$

**Table 9:** Non-linear optical parameters of LAM molecule.

NLO property	LAM	Standard reference material urea
Dipole moment (μ) (Debye, D)	4.41	2.37 [63]
Linear polarizability (α)	6.78 × 10^−24^	4.23 × 10^−24^ [80]
Anisotropy of polarizability Δα (esu)	1.83 × 10^−23^	5.666 × 10^−24^ [81]
First-order hyperpolarizability (β) (esu)	6.81 × 10^−31^	3.7 × 10^−31^ [63]
Second-order hyperpolarizability (γ) (esu)	1.14 × 10^−38^	4.16 × 10^−36^ [82]

The anisotropy of polarizability Δα = $\frac{1}{\sqrt{2}}\sqrt{{\left(\alpha_{xx}-\alpha_{yy}\right)}^{2}+}{\left(\alpha_{yy}-\alpha_{zz}\right)}^{2}+{\left(\alpha_{zz}-\alpha_{xx}\right)}^{2}+6\alpha_{xx}^{2}$.

(41) First−orderhyperpolarizability,β=(βx2+βy2+βz2)12

where $\beta_{x}=\beta_{xxx}+\beta_{xyy}+\beta_{xzz},\beta_{y}=\beta_{yyy}+\beta_{yxx}+\beta_{yzz}\;\text{and}\;\beta_{z}=\beta_{zzz}+\beta_{zxx}+\beta_{zyy}$.

Second order hyperpolarizability (nonlinear induced polarization per molecule),

(42) $$\gamma =\frac{1}{5}\left(\gamma_{xxxx}+\gamma_{yyyy}+\gamma_{zzzz}+2\gamma_{xxyy}+2\gamma_{xxzz}+2\gamma_{yyzz}\right)$$

The dipole moment (μ) of LAM molecule (μ = 4.41D) appears to be 1.86 times than that of the ideal reference material urea (μ = 2.373D) (Table 8). The β value of LAM molecule (β = 6.81 × 10^−31^ esu) has turned out to be 1.84 times than that of urea (β = 3.7 × 10^−31^ esu) (Table 8). The value of α depends on the longitudinal components of α_xx_, α_yy_, and α_zz_. Similarly, the value of the longitudinal components of β_xxx_, β_xzz_, β_yzz_, β_zzz_, β_zxx_ and β_xyz_ are the largest. Dominance of these components over others creates greater delocalization of charges in these directions. The component β_xyy_, β_yyy_ and β_yxx_ along their directions are relatively average in value and in the direction of β_zyy_ the component value is the lowest. Such behaviour causes optical nonlinearity in the molecule. The non-zero value of dipole moment and high β value proves that LAM molecule is polar in nature and gives explanation for the microscopic origin of NLO activity in LAM crystal.

The band gap of the LAM molecule has been measured as 5.03 eV from HOMO-LUMO analysis. This value is compatible with the band gap value obtained from the UV–vis data (5.00 eV). There is a small difference between theoretically and experimentally measured value as the theoretical computations have been performed on single molecule in the gaseous phase, on the other hand, the experimental data had been collected from real life three-dimensional solid phase where the van der Waals force and crystal field enormous contribution on the molecules and thus affecting its properties [65,83].

## 6 Conclusions

Transparent and colourless crystal of LAM has been successfully harvested by slow evaporation solution method at room temperature. From powder X-ray diffraction analysis and by Rietveld refinement, the crystalline planes, lattice parameters were obtained properly and it revealed orthorhombic crystal system. From the strain analysis using Hall–Williamson's equation, the existence of compression due to some defects is evident. Morphology of the grown crystal reveals a higher growth rate along the c axis. SEM photographs and EDAX analysis demonstrate the layer-like growth pattern and stoichiometric ratio of the constituent elements of the crystal. The existences of the functional groups and their corresponding vibrations have been validated by FTIR analysis. The UV–vis spectra demonstrate excellent optical transmittance along whole visible spectrum, which is required for NLO application. The small value of Urbach tail energy indicates good crystalline perfection. The predicted nonlinear refractive index n_2_ and nonlinear susceptibility χ^(3)^ are high in value, indicating its potentiality as NLO crystal. The dielectric property has been studied and the value of α has been measured revealing its good polarizable nature. Band structure calculation reveals an insulating system for LAM crystal. The bottom of the CB and top of VB are largely due to 2p orbitals of O, N and C atom. In addition, HOMO-LUMO energy gap and MEP mapping had been achieved by quantum chemistry computations, from where, a little variation in band gap energy is observed between theoretical and experimental results. The HOMO level was mainly sited on the π-system of carboxyl and amino group of LAM. The value of HOMO-LUMO energy gap for LAM molecule indicates polarizable nature, thus suitable for UV and deep UV NLO applications. The value of μ and β proved to be 1.86 and 1.84 times than that of urea (standard reference material). In general, the study proves that quantum chemical computations on amino acids provide the correct prediction of numerous electrostatic NLO properties giving reliance in using DFT methods to investigate the NLO properties of complex molecules.

## CRediT authorship contribution statement

**Md Anisur Rahman:** Writing – original draft, Software, Methodology, Investigation, Formal analysis, Data curation. **Jiban Podder:** Writing – review & editing, Visualization, Validation, Supervision, Methodology, Investigation, Conceptualization.

## Data statement

The data presented in the paper are not available in the internet but obtained through experimental investigations in the lab.

## Funding

This research work has not received any financial assistance from commercial, public or not-for-profit organization.

## Declaration of competing interest

This is to certify that this manuscript does not make any conflict of interest with any person or Institution or laboratories or any work. This manuscript is not considered for publication elsewhere.
